# Insights into the HIV-1 Latent Reservoir and Strategies to Cure HIV-1 Infection

**DOI:** 10.1155/2022/6952286

**Published:** 2022-05-31

**Authors:** Ruojing Bai, Shiyun Lv, Hao Wu, Lili Dai

**Affiliations:** ^1^Center for Infectious Diseases, Beijing Youan Hospital, Capital Medical University, Beijing 100069, China; ^2^Beijing Key Laboratory for HIV/AIDS Research, Beijing 100069, China

## Abstract

Since the first discovery of human immunodeficiency virus 1 (HIV-1) in 1983, the targeted treatment, antiretroviral therapy (ART), has effectively limited the detected plasma viremia below a very low level and the technique has been improved rapidly. However, due to the persistence of the latent reservoir of replication-competent HIV-1 in patients treated with ART, a sudden withdrawal of the drug inevitably results in HIV viral rebound and HIV progression. Therefore, more understanding of the HIV-1 latent reservoir (LR) is the priority before developing a cure that thoroughly eliminates the reservoir. HIV-1 spreads through both the release of cell-free particles and by cell-to-cell transmission. Mounting evidence indicates that cell-to-cell transmission is more efficient than cell-free transmission of particles and likely influences the pathogenesis of HIV-1 infection. This mode of viral transmission also influences the generation and maintenance of the latent reservoir, which represents the main obstacle for curing the infection. In this review, the definition, establishment, and maintenance of the HIV-1 LR, along with the state-of-the-art quantitative approaches that directly quantify HIV-1 intact proviruses, are elucidated. Strategies to cure HIV infection are highlighted. This review will renew hope for a better and more thorough cure of HIV infection for mankind and encourage more clinical trials to achieve ART-free HIV remission.

## 1. Introduction

Over 70 million people have been infected with human immunodeficiency virus 1 (HIV-1) so far since the first outbreak of the HIV-1 epidemic [1] in 1981, and since then, millions of survivors have lived with HIV-1 who are the beneficiaries of antiretroviral therapy (ART). The 2019 UNAIDS Report and World Health Organization both estimate that there are 38~70 million people living with HIV-1 infection. Of those individuals, almost 25 million have access to antiretroviral therapy (ART). Various studies have shown the half-life of the HIV-1 reservoir can range somewhere between 44 months and 13 years, and in some cohorts, no decay was observed at all. Thus, lifelong ART is required to maintain viral suppression and achieve the best health outcomes in the majority of individuals [2]. Nowadays, a number of evidence has pointed out that the risk of recurrence is related to the latent reservoir (LR) of HIV-1, also known as HIV latency, which is a pool of resting CD4+ T cells infected with replication-competent proviruses in patients treated with ART. These infected cells have stopped generating new viral particles temporally or for a long time since the treatment. Nonetheless, these infected memory CD4+ T cells which permit HIV-1 to escape from immune surveillance are the main obstacle to HIV elimination. Thus, using ART treatment to eliminate HIV is currently unrealistic.

At present, the eradication of HIV is still in need of accurate quantification of the HIV-1 LR. Although a barrage of improved assays for measuring the HIV reservoir size has been developed, there is no broad consensus on the methodology yet. Despite more than three decades of efforts, the understanding of the HIV-1 latent reservoir is not enough, and to have more understanding of it is the priority before thorough elimination of it can be achieved (a cure) and plasma viremia can be persistently inhibited after ART withdrawal (a functional cure) (Figure 1). In this review, the definition, establishment, and maintenance of the HIV-1 LR are elucidated, and standard and state-of-the-art approaches to quantify reservoir size are reviewed. Finally, current progress of the elimination of the HIV LR is highlighted.

On the left is the ART intervention on HIV-1 virus with recurrent infection after HIV-1 LR measurement to eliminate HIV-1. On the right is the strategy of eliminating HIV-1 LR carried out by persistence in long-lived memory T cell and homeostatic promotion of T cells.

## 2. Definition of HIV-1 LR

The HIV-1 LR is defined as a small pool of latently infected cells that persist for decades in people living with HIV (PLWH) who have received ART [3]. These cells harbor integrated and intact proviruses that do not actively produce infectious virions but can do so upon stimulation [4]. Although such cells are extremely rare (around 1 in 1 million resting CD4+ T cells), the reservoir is long-lived, with an estimated half-life of 44 months [5]. This indicates that ART alone will not eradicate the reservoir in a lifetime.

The precise nature of the HIV-1 LR remains unclear. The assessment of the transcriptional and translational status of persistent HIV proviruses in virally suppressed individuals challenges our definition of HIV latency. Whereas viral latency is often associated with transcriptional latency (i.e., the lack of transcription from the HIV promoter), an increasing number of studies have indicated that complete silencing of the HIV promoter is a rare event. Therefore, a relatively large fraction and possibly the majority of latently infected cells (cells that do not produce viral particles) may express low levels of short viral transcripts [6]. Although these abortive transcripts are frequently produced, they rarely elongate enough to generate complete or spliced transcripts [7]. Accordingly, the production of viral proteins by latently infected cells appears to be rare [8].

### 2.1. Establishment of the HIV-1 LR: When, Where, and How

#### 2.1.1. When

The current consensus is that the reservoir is established in individuals immediately after HIV-1 infection and even on early ART [9]. Animal experiments show that HIV-1 LR stays in lymph nodes (LNs) and gut-associated lymphoid tissues (GALTs) within the first 72 h of mucosal simian immunodeficiency virus (SIV) infection [10]. Also, the HIV-1 LR was established in less than 10 days in a unique case who initiated preexposure prophylaxis/ART as long as 10 days after infection, and he experienced viral rebound 225 days after ART withdrawal [11]. The exact time of HIV-1 LR establishment in humans remains unclear.

#### 2.1.2. Where

In the case where ART is not administered, the stimulated CD4+ T cells serve as the main target of HIV infection and die rapidly [12]. Only a minute fraction of these infected cells survive and become a long-lived reservoir of latently infected cells [13]. However, peripheral T cells only account for less than 2% of the total cells infected, so circulating T cells are not a unique site of HIV replication and are unlikely to represent the most favorable environment for the establishment of HIV latency. In the presence of ART, these reservoirs are particularly spread in GALTs and LNs [14] relative to the spleen, liver, lung, central nervous system, and bone marrow [15]. Lymphoid tissues may especially represent a favorable environment for the establishment of viral latency. It is not surprising that HIV-infected cells are found in multiple tissues after years of ART [16].

Currently, imaging the persistent tissue reservoir in living people on ART is not possible. Recently, a study of tissues collected from 6 postmortem PLHIV patients revealed that HIV proviruses existed in all 28 tissues examined wherein the blood and the lymphoid system serve as the main vectors for virus dissemination throughout the body [16]. Besides, HIV-1 DNA is highly enriched in CD4+ tissue-resident memory T (TRM) cells in the female genital tract (particularly the cervix) [17] and the male genital tract which may be a tissue reservoir where macrophages are enriched [18]. Macrophages enriched in these tissues may serve as potential viral sanctuaries. However, whether reproductive tracts are tissue reservoirs remains poorly understood.

#### 2.1.3. How

There are two models for the establishment of the HIV-1 LR. First, as CD4+ TRM cells are the predominant population [12], the activation-to-quiescence transition using a defined cocktail of cytokines, including tumor growth factor-beta (TGF-*β*), interleukin-10 (IL-10), and IL-8, probably provides an opportunity for the establishment of HIV latency and allows the persistence of latently infected cells [19]. In the immune microenvironment, checkpoint molecules expressed on T cells are the immunosuppressive factors that significantly repress T cell activation and contribute to HIV-1 latency, of which PD-1, LAG-3, and TIGIT are the known markers to block HIV-1 persistence during ART [20–22]. More studies have explained the active role of PD-1 that blocks HIV transcription [23, 24]. Of note, the coculture of monocytes or myeloid dendritic cells (mDCs) with activated HIV-infected T cells augments the transition to a postactivation state of latency, indicating the potential cell-to-cell contact during the establishment of HIV latency [25, 26].

The two means for the establishment of viral latency consist of direct infections in CD4+ TRM cells and cell-to-cell transmission between infected and uninfected CD4+ TRM cells. Although the inefficient infection in CD4+ TRM cells can be blocked during the HIV replication cycle, the indirect cell-to-cell transmission gives way to HIV-1 latency [27]. Besides, soluble factors are also contributors to HIV-1 latency in resting CD4+ T cells. For instance, IL-7, for T cell homeostasis, regulates the activity of the restriction factor SAMHD1 and exacerbates the vulnerability of CD4+ TRM cells to HIV-1 [28, 29]. Similarly, the chemokines CCL19 and CCL20 participating in cell trafficking from other tissues to LNs and GALTs may increase the possibility of HIV infection in CD4+ TRM cells via modifying the actin cytoskeleton to allow the nucleus of HIV-1 DNA to enter a LR of quiescent integrated HIV-1 DNA [30]. The sites of CD4+ TRM cell recruitment may impact HIV-1 susceptibility: CD4+ T cells derived from lymphoid organs (the spleen and tonsil), subjected to moderate-level activation, benefit from the establishment of the HIV LR [31].

## 3. Maintenance of the HIV-1 LR

Several studies over the past decade have reported that such clonal expansions of latently infected cells—the duplication of partial and near-full-length HIV genomes and/or integration sites—are the key mechanism of maintenance of the HIV reservoir [32–34]. The infected cells in clones in samples of patients undergoing ART may differ from each other [35]. The following mechanisms explain the heterogeneity [36]: (a) antigen-driven clonal proliferation of infected cells [37], (b) homeostatic proliferation of infected cells [38], and (c) HIV integration-induced cell proliferation [39]. Although the first mechanism is a major driver of the maintenance of the HIV reservoir as confirmed by most researchers, the effect of the coexistence of the other two mechanisms cannot be excluded [36, 40]. Therefore, clonal expansion of latently infected cells contributes to the maintenance of the HIV-1 LR.

## 4. Measurement of the HIV-1 LR

Despite clinically efficacious ART, replication-competent HIV-1 persists as latent proviral DNA capable of rekindling viral replication after ceasing ART. Therapies to eliminate latent HIV-1 are being developed for a complete cure. Accurate assays to quantify intact or rebound-competent HIV-1 are critical to this effort. Four challenges obstruct the precise quantification of the HIV-1 LR. The gravest one is that in ART-treated PLWH with mutations and/or deletions, HIV-1 proviruses produce defective mutants which are unable to replicate. However, not all intact genomes (without defective mutations or deletions) can produce virions after induction. It is more of an occasional incidence of latently infected cells. Finally, most HIV reservoirs that reside in tissues cannot be accurately sampled with current specimen-collection approaches [41–44].

The conventional quantification of HIV, the gold standard VOA assay, can merely detect the transcribed replicates of totiviruses; therefore, this technique underestimates reservoir levels. However, PCR analysis for total HIV DNA or Alu-Gag PCR also quantitates a large amount of defective HIV DNA fragments and thereby overestimates reservoir levels. Bruner et al. developed a new method, the intact proviral DNA assay (IPDA), to amplify HIV *ψ* fragments and the Env gene using droplet digital PCR (ddPCR). HIV DNAs used for the amplification of *ψ* are limited to those whose 3′ ends are defective, and only the DNAs used for the amplification of Env have defective 5′ ends. Double-positive HIV DNA amplified using IPDA is intact HIV DNA, which not only corroborates the results from the VOA assay but also compensates for the flaw of the PCR assay that can yield false-positive results due to defective viral fragments. Based on these studies, reservoirs of potential intact HIV DNA and those of defective HIV DNA hold completely different traits and effectively overcome the three challenges mentioned above (the fourth challenge is an objective existence).

IPDA for HIV DNA quantification using ddPCR targets multiply regions of proviral DNA to exclude deleted and hypermutated proviruses. The ddPCR is the third-generation PCR technique, which partitions samples into 20,000 droplets, and each droplet contains an independent reaction system and tremendously reduces interference from background nucleic acid molecules during PCR amplification. Therefore, it is competent in the quantification of low-copy nucleic acid molecules of interest. The ddPCR technique uses the ratio of positive to negative droplets among the 20,000 droplets to calculate the copy number of target nucleic acid molecules, without the use of standard substances for standard curves. Here is the specific principle: an amplicon is added at the packaging signal and the conserved site in the env sequence, respectively, excluding 90% of deficiency; at the same time, a mutant protein is added to bind to the amplified loci of env, excluding 95% of most frequent mutations. As a result, double-positive DNA fragments can be identified as intact proviral DNA. Meanwhile, two amplicons with the same distance as that of the reference RPP30 gene in another hole are designed for shearing, control (the strand break of DNA between two amplicons during DNA extraction will reduce the double-positive number detected and there by the results could be underestimated), and cell quantification. By this means, the size of reservoirs can be calculated.

IPDA is optimal for high-throughput analysis in large interventional or observational clinical studies. For instance, a recent longitudinal cohort analysis has evaluated the decay rate of intact and defective proviruses in a large number of patients by using this technique [45]. Another study using this measurement found no relationship between heroin or cocaine use and the reservoir size [46]. This technique offers competitive advantages of 97% elimination of defective proviruses, only about 1.5-fold overestimation of the LR size, simpler operation, lower cost, and greater speed than traditional QVOA. Nonetheless, sequence polymorphisms in some patients, the requirement for alternative primers or proteins, and within-clade diversity dependence obstruct the efficient amplification so the provirus inducibility cannot be accurately quantified.

## 5. Elimination of the HIV-1 LR

### 5.1. Strategies Targeting the HIV-1 Replication Cycle

#### 5.1.1. Early ART

Early initiation of ART is aimed at reducing virus diversification since the diagnosis of HIV infection can prevent damage of immune function as much as possible, minimize HIV-related complications in treated individuals, and prevent human-to-human transmission by lowering viremia [47]. Early ART initiation currently cannot achieve an HIV cure in adults or mothers; however, the infants can be the beneficiaries of the early interventions. As these early interventions reshape the association between the virus and the immune system, HIV infection can be ultimately controlled after ART withdrawal in a certain proportion of patients that have received ART at an early stage. This population accounts for approximately 5–10% of all HIV-infected individuals, who become posttreatment controllers achieving ART-free viral remission [48, 49].

During long-term ART, much of the reservoir derive from the cells that are infected just before treatment initiation. It is arguable that in the preintervention period, the putative reservoir is unstable [50, 51]. This implies that during early ART, the rapidly changing immune environment shifts the balance toward a state in which HIV latency can be achieved. Presumably, the massive reduction in HIV-1-associated inflammation and T cell activation reduces the turnover of the reservoir, leading to the generation of longer-lived cells harboring intact genomes. Immune stimulation under the cover of ART (preferably with the coadministration of a therapy that induces the killing of infected cells) might work best during this window of opportunity.

#### 5.1.2. Transplantation

There are two studies of two patients (from Berlin and London) who underwent allogeneic stem cell transplantations from CCR5132/132 donors who achieved an HIV-1 cure. After monitoring their plasma viremia for 10 and 2 years, respectively, negative results were found after ART withdrawal [52, 53]. These studies reported the depletion of the HIV-1 LR during pretransplant conditioning, and the reservoirs were replaced with donor cells with Delta 32 CCR5 deletion to confer resistance to R5-tropic HIV-1 infection [54]. As there are a lack of CCR5132/132 donors, diagnosis delay of HIV infection in most cases, and massive expenditure, HIV cure for most patients is unrealistic. Therefore, silencing, the basic principle of HIV-1 cured, or HIV-1 LR elimination is the priority.

#### 5.1.3. Gene Editing

Recent years have seen the emergence of several gene editing tools, such as CRISPR Cas9 and zinc-finger nucleases (ZFN). These techniques are potent in enhancing host resistance or disrupting viral latency through the silencing of integrated provirus in the host, which paves the way for an HIV-1 cure. These strategies offer the precise correction of sequences in a genome. Different from LRAs, they can produce desired outcomes without a physiological impact throughout the body. Notably, as several studies reported off-target effect, the safety of these methods must be evaluated before the clinical application. [55] So far, the only clinical study has achieved Delta 32 CCR5 deletion using ZFN-targeted editing to help patients gain partial genetic resistance to R5-tropic HIV-1 infection [56]. Most studies focus on the efficacy of CRISPR-Cas9 because of its simple operation. Some studies have performed CCR5 or CXCR4 ablation in CD4+ TRM cells using CRISPR-Cas9 to protect cells against CCR5 or CXCR4 tropic HIV-1 infection [57–59]. To specifically knockout or silence the HIV-1 proviral genome, which is the premise of HIV-1 LR elimination, is feasible with CRISPR Cas9 therapy [60, 61]. Besides, by targeting other domains of the HIV-1 proviral genome, the resultant indels in these domains introduced by NHEJ-mediated repair can result in frameshift mutations to deactivate the provirus [62, 63]. This strategy, in combination with a novel drug delivery system, was successfully performed in mouse models [64]. During the viral replication cycle, though multiple editable sites can be targeted in the HIV-1 proviral genome using a CRISPR-Cas9 strategy, therefore, more options for quasispecies diversity are provided; the lack of adequate viral vectors or lipid compounds is a barrier to effective delivery [65]. Considering that there is a substantial number of LNs, GALTs, and other tissues with HIV-1 LR, the elimination of the reservoirs is a project that has to be exerted with such great effort that current strategies can hardly make it.

#### 5.1.4. Shock and Kill

The shock and kill strategy was put forward by Siliciano and Deeks in 2012. It is a combination strategy using latency-reversing agents (LRAs) in immunotherapeutic treatment (e.g., T cell vaccines) to shock and kill intervention activated cells via reactivating them, thereby reducing the size of the LR and preventing viremia rebound [66, 67]. Since the single use of either constituent merely shows limited clinical benefit, the combination strategy is yet to be tested, leaving its efficacy to be in doubt. However, its flaws are currently known as toxic side effects and systemic immune response alongside HIV-1 latency reversal.

The commonly used LRAs can be assigned to six groups by pharmacological mechanisms: histone posttranslational modification modulators, nonhistone chromatin modulators, NF-*κ*B stimulators, TLR agonists, extracellular stimulators, and a miscellaneous category of unique cellular mechanisms [68]. The nonspecific histone deacetylase inhibitors (HDACIs) characterized to acetylate the histone of integrated proviral promoters in vitro are the most prominent at present. Clinical trials for the promising HDACI candidates, including vorinostat, disulfiram, and romidepsin, reported that these HDACIs effectively induced viral replication and killed activated cells harboring HIV once the immune system was activated [69–71].

Inspired by a current finding that some of the latently infected CD4+ T cells are HIV-specific, efforts have been made to develop cost-effective and safe HIV-specific vaccines to reverse HIV latency [72, 73]. HIV vaccines reactivate HIV-specific latently infected cells to eliminate them via stimulated cytotoxic T lymphocytes (CTLs) [74], thus offering a near-complete representation of viral quasispecies and an enhanced killing effect of the shock and kill strategy [67]. The shock effect can be enhanced using a latency-reversing intervention with the involvement of other immune cells. For instance, GS-9620 (a TLR-7 agonist) can reactivate HIV-infected CD4+ TRM cells probably through IFN-*γ* release from plasmacytoid dendritic cells [75]. Despite those reported effective results, some studies had inconsistent results and reported that these strategies have nonsignificant effect on diminishing the size of the HIV reservoir in patients [76, 77]. Some studies even reported adverse effect on immune response after the administration of these strategies [78, 79]. Some scholars from the University of Pennsylvania proposed that the research and development of COVID-19 vaccine will help promote the research and development of HIV vaccine. These undesirable results may be ascribed to insufficient killing effect, so extensive studies using strategies with improved killing effects are being developed, including employing broadly neutralizing antibodies and immune checkpoint inhibitors [80], as shown in the details below.

#### 5.1.5. Block and Lock

There are some data indicating that the HIV genome that becomes preferentially enriched in intergenic regions becomes hypermethylated over time through multiple mechanisms, resulting in less HIV expression [31]. This evolution of proviral distribution reflects the survival of cells with defective HIV viruses and that of the viruses in regions of the genome that promotes “deep latency.” A relatively novel cure strategy, namely, block and lock, by contrast, aimed at reinforcing latency (“block”) rather than inducing latency reversal, has been proposed to prevent viremia rebound following ART discontinuance [81, 82]. To illustrate it in detail, transcriptional gene silencing (TGS) by promoter targeting small interfering RNAs (siRNAs) can rapidly recruit chromatin remodelers to repress HIV-1 transcription [81]. To enhance or maintain the HIV-1 latency, the targeted inhibition of the HIV-1 positive regulator Tat is employed so that the viral replication cycle can be blocked (“lock”) at the transcriptional level [82]. Clinical studies about other potential HIV-silencing techniques are in progress. Among the potential candidates, inhibitors of mammalian target of rapamycin (mTOR) have been justified as effective [83]. Their therapeutic efficacy and safety have been validated in clinical studies.

Though the efficacy of “shock and kill” approach is uncertain, evidence has pointed out that it can remarkably diminish the LR size and is expected to achieve ART-free HIV remission.

#### 5.1.6. Strategies That Target the Immunity

*(1) Therapeutic Vaccination*. Therapeutic vaccination enhances the host immune response to HIV-1, thus eradicating the HIV-1 LR or diminishing viremia rebound as a cure. This way leverages vaccine inoculation during sustained ART-mediated viral suppression. During ART interruption, the time to viral rebound, the size of the LR, and the profile of the host immune response are detected to confirm the efficacy of HIV-1 vaccination.

HIV-1 vaccines only trigger narrow CTL response to specific HIV-1 proteins (e.g., gag) after inoculation. CTL escape mutants can be enhanced due to a weaker efficacy since the mutation happens during primary infection [84, 85]. Therefore, HIV-1 vaccine is seemingly more reliable as it triggers a broader anti-HIV-1 immune response. Some researchers stated that they would fabricate dendritic cell- (DC-) based vaccines using autologous DCs cocultured or transfected with inactivated HIV-1 to stimulate CD4+ TRM cells to boost immune responses [86, 87]. Interestingly, a study reported that a combination of HIV-1 vaccines and Tat-based immunization, a “block and lock” strategy, continually suppressed the proviral reservoir followed by the recovery of immune function. This suggests that therapeutic vaccination can boost the immune response in HIV-1 infection clearances [88].

Currently, HIV-1 vaccines have not yet induced sustained HIV-1 remission. Among these studies, a study by Davenport et al. expressed their concern that although the most efficacious vaccines could block 80% of viral reactivation, viremia rebound could quickly occur in these patients in less than five weeks after ART withdrawal [89]. This indicates that HIV-1 vaccination cannot thoroughly eliminate the latent HIV-1 reservoir, which means it is insufficient to overcome viral rebound and further cure HIV-1 infection. To make up for this shortcoming, in contrast to using HIV-1 vaccination separately, a proper combination of strategies, such as shock and kill, targeted to suppress viral rebound can be more effective in the treatment. Two clinical studies have adopted and validated this combination protocol (gag-based vaccination followed by HDCAI latency reversal); however, plasma viremia has been redetected in less than two weeks after that [90, 91].

#### 5.1.7. Broadly Neutralizing Antibodies (bNAbs)

Immunotherapies are popular as the HIV antagonists directly target cells expressing the HIV envelop proteins that interact with the lymphocyte cell-surface molecule CD4 so the latent HIV reservoir can be eliminated. Some studies reported that bNAbs targeting specific envelope glycoproteins probably suppress virus replication in vivo [92, 93] by blocking the entry and spreading of virus. Theoretically, bNAbs can trigger host-mediated cytotoxicity by binding themselves to envelope proteins expressed on the surface of infected immune cells that have already been stimulated, thereby reducing the active reservoir. Whether the infected cells are killed in vivo remains unproven, though indirect evidence suggests that it may have some effect [94].

Some early proof-of-concept studies about several strategies aimed at enhancing PTC were being completed. Even if bNAbs cannot directly clear the latent cellular reservoirs of HIV infection, it has been postulated that they achieve this for highly immunogenic antibody-antigen response and thus might stimulate potent HIV-specific immune response and achieve post-ART control [95].

Hindered by the barriers to HIV-1 vaccine development and HIV-1 eradication and remission, passive transfer of monoclonal HIV-1 neutralizing antibodies is another option. The small-molecule drugs bNAbs featuring longer half-lives currently being used not only have an attractive price but also stimulate the immune response directly and exert a robust killing effect on the latently infected cells. By this means, the course of HIV-1 infection can be shortened. As of now, several clinical trials have used various bNAbs and successfully verified the efficacy of suppressing and controlling viremia rebound [96].

#### 5.1.8. Chimeric Antigen Receptor T (CAR-T) Cells

CAR-T cell therapy has been employed to treat B cell malignancies [97–99], and there is evidence that reveals its potential in treating HIV-1 infection. For eliminating latently infected cells, autologous T cells can be engineered to express a unique CAR to confer HIV-1 antigen specificity. Patients who receive CAR-T cell therapy can directly raise the CTL response to cells expressing the disease epitope [100], so CAR-T cell therapy can eliminate latently infected cells with HIV-1-associated antigen through the killing effect of CTLs, aiding in the control of the virus without ART. Some in vitro experiments using CAR-T cell therapy have ascertained a satisfactory efficacy of anti-HIV-1 CAR-T cells [101, 102]. An animal experiment based on mouse models where the mouse cells were infected with HIV-1 showed the effective eradication of HIV-1 infected cells [103]. Notably, preclinical studies ascertained that bNAb-based CAR-modified CD8+ T cell therapy is possible as a cure; however, it needs to be validated by high-quality clinical studies. At present, CAR T-cell therapy is flawed with CAR T cell expansion, persistence, off-target effect, and severe cytokine release syndrome (sCRS). More work is needed to address these issues.

#### 5.1.9. Immune Checkpoint Blockers

The definition of immune checkpoints is a large sum of regulatory pathways that potently suppress the immune activity, particularly the T cell activity; the associations between immune checkpoints, immune exhaustion, and impaired function have been proven (reviewed by Wykes and Lewin) [104]. CD4+ T cells in the peripheral circulation and lymphoid tissues express high levels of immune checkpoint markers, including programmed cell death protein 1 (PD-1), cytotoxic T lymphocyte antigen 4 (CTLA-4), and other markers that adhere to the membrane to exert the killing effect on HIV once activated [22, 105, 106]. Expressions of immune checkpoints are upregulated in HIV-specific CD4+ and CD8+ T cells when HIV-specific immunity is activated in untreated and treated cases and ex vivo. The single or combined use of antibodies against these markers can enhance the upregulation [21]. In this way, the HIV LR can be reduced [104]. The upregulated checkpoints in latently infected T cells incorporate PD1/PD-L1 and CTLA-4 as the main components. These markers are worthy of research on drug delivery or HIV-1 clearance [107–109]. In vitro studies on the efficacy of immune checkpoint blockers claimed that the HIV-1 LR could be inhibited via the IC-mediated manner, and in vivo studies also confirmed its effect of promoted latency reversal. These results show the anti-HIV-1 potential of immune checkpoint inhibitors [23, 24, 110].

## 6. Combination Therapy for HIV-1 Infection

At present, no single treatment can eliminate HIV-1 LRs, nor even remission. Combination strategies can minimize the LR level with the host immune system defending against latent infection efficiently after treatment. Most ongoing studies on HIV-1 cures designed to assess their safety and relevant mechanism remain in preclinical and transitional phases. Clinical trials for assessment of combination approaches are getting more and more attention [111], and more efficacious combination strategies are expected to achieve a complete cure or remission [91, 112].

## 7. Conclusions

Some progress in HIV-1 cure development has been made, such as reduced HIV-1 mortality and HIV-1 LR measurement. But there is still a long way to go for the research and development of HIV-1 elimination and remission as preexisting measurement cannot guarantee 100% accurate quantitation of the HIV-1 LR at each stage, and current therapies cannot achieve complete clearance due to the persistent LR.

The past decade has witnessed many strategies proposed as a cure, among which the shock and kill therapy is the most promising. Validation studies of the shock and kill strategy reported neither decrease nor increase in the time to viral rebound, and the virus reactivation still existed in vivo. Hence, the enhancement of the killing effect against the HIV-1 LR and alternative methods, such as therapeutic vaccination and immune boosters against HIV-1 infection via augmenting immune-mediated control of HIV-1 after ART withdrawal, is required. Regarding novel methods, such as immune checkpoint inhibitors, gene editing tools, and CAR-T cell therapy, their efficacy needs to be verified in more clinical studies. These approaches have renewed hope for an HIV-1 cure. Posttreatment complications, such as adverse effects weakening immune response, pose challenges in patient compliance and precise assessments of the therapeutic efficacy. The complexity of LR quantification is associated with the inherent variability of the HIV-1 genome, the low incidence of latently infected cells, and the abundance of defective proviruses.

Instead of emphasizing on single-agent strategies, the combined use of synergistic anti-HIV-1 agents (e.g., LRAs plus HIV-1 vaccination) is more likely to remarkably reverse the HIV-1 LR and achieve the ultimate goal of long-term ART-free viral remission.

## Figures and Tables

**Figure 1:** HIV-1 LR measurement and elimination strategy.
